# Construction of a Hybrid Teaching Model System Based on Promoting Deep Learning

**DOI:** 10.1155/2022/4447530

**Published:** 2022-01-28

**Authors:** Yingjie Sun, Yang Li, Yuan Tian, Wanqiang Qi

**Affiliations:** ^1^Aviation University of Air Force, Changchun, Jilin 130022, China; ^2^School of Automotive Engineering, Jilin Teachers Institute of Engineering and Technology, Changchun, Jilin 130022, China

## Abstract

The rapid development of computer network technology in today's society has also brought new opportunities for the transformation of the teaching management mode of colleges and universities. Nowadays, most colleges and universities are gradually improving the construction of campus informatization projects, further integrating school teaching resources, centralizing the work related to the work process, and carrying out platform management to improve the daily work efficiency of various departments of the school, which is also prominent from the user experience. Humanized management out of school. This paper designs and develops a set of online teaching management system suitable for colleges and universities, realizes the informatization of college teaching management, and solves the traditional teaching methods, such as the inability of offline correspondence students to take classes in time and the limited teaching venues. Through comparison and analysis, in order to ensure that the system has better portability, this article will mainly adopt the MVC architecture model to develop and design the entire school hybrid teaching management system. The MVC architecture model is mainly developed based on the abstract design model. Strong reusability, combined with the system architecture, the main choice for database selection is development based on Oracle database technology. In the specific development process, the detailed business requirements and functional requirements of the entire school online teaching management system will be analyzed in detail. Based on this, by adopting an object-oriented approach, the system management included in the school's hybrid teaching management system will be further analyzed. Detailed analysis and design of the specific functional structure, work flow, work sequence diagram and class diagram of the online learning management and article management functional modules, and finally complete the implementation and testing of the various functional modules of the system.

## 1. Introduction

At present, computer technology and Internet technology have been integrated into all corners of society, greatly affecting and changing our production and lifestyles, and providing people with great convenience. From the time when the Internet was underdeveloped to the present, the convenience of Internet technology has affected all walks of life. Among them, education is a national priority and key development business, and informatization has also been applied early in education. Educational information The concept of chemistry has also begun to be widely recognized and valued. In recent years, with the continuous improvement of my country's education level, some schools have begun to use information management systems in order to provide their own management and teaching levels. According to their own teaching management characteristics, they have designed and developed a series of education information management platforms to promote teaching Management work is developing in the direction of informatization. The emergence of a networked hybrid teaching management system has brought major reforms to the hybrid teaching management, informatization construction, sharing and release of teaching resources, networked educational administration and comprehensive management of student information in colleges and universities, and many colleges and universities have burst out The new teaching management ideas are all benefited from the rapid development of networking and informatization. As a brand-new management method, the hybrid teaching management system is an important application of computer technology in the field of education. It strengthens the comprehensive management of schools, improves the efficiency of teachers, and advances the process of university management. At present, from a technical perspective, the current teaching management system used by private training institutions is mainly based on the C/S architecture. This architecture is simple in structure and easy to develop. The internal staff of the training institution can complete the development or commission small software The development work is done on behalf of the development, generally the cost is low, and it is widely used in small training institutions. For colleges and universities, C/S architecture is usually difficult to meet their needs, and they mostly use teaching management systems based on B/S architecture. The B/S architecture system is more difficult to develop than the C/S architecture, but it has more powerful functions and is more suitable for school use scenarios. The B/S structure system is easy to maintain, which is conducive to the expansion of the school. On the other hand, the B/S architecture adopts a modular system architecture, and the internal modules of the system are loosely coupled, which facilitates the expansion of the department and the increase of system functions, and is more suitable for changes in the teaching management business of colleges and universities. According to the school's mixed teaching management business needs and the needs of information construction, it is very necessary to design and develop an information management system suitable for the school's own development. Through the design and implementation of this system, it can not only improve daily work and student management Efficiency, but also can reduce costs, improve their own competitiveness, and better provide students with a good learning environment and conditions.

## 2. Related Theoretical Methods

### 2.1. MVC Architecture

The whole university hybrid teaching management system mainly adopts the object-oriented design method for development and design. Through comparison and analysis, the system architecture design selection is based on the MVC (Model View Controller) architecture method. Through the use of MVC The architecture system can effectively improve the scalability and maintainability of the system. At the same time, the code reusability can be further improved in the system development process, which is convenient to reduce the system development cycle and the development cost can also be reduced. The specific situation of the relationship between the layers of the entire MVC architecture is shown in Figure 1.

The entire MVC architecture is mainly composed of three parts: view, model, and controller. Among them, the view part is mainly able to provide system users with a human-computer interaction interface, which can collect user specific operations, and can also display the content processed through the model layer. Normally, the view part is usually made of HTML elements. With the continuous development of computer technology, this module can be used to query the status of the model part and check the status change of the controller module. With the continuous development of computer technology, in order to be able to continuously enrich the machine interaction operation, provide users with more convenient and efficient interaction Experience, XML and Flash and many other elements are being applied. The model part is used to process various different types of data according to certain logic. This module can be used to query the status of the view part. In order to effectively improve the processing capabilities of various types of data, usually one model can be combined with multiple view blocks. Correspondence and processing. The controller part is the most core part of the entire MVC architecture. It can coordinate the information interaction between the view part and the model part, and process the user time information fed back by the view module to ensure the stable and reliable operation of the system. Combined with the MVC architecture diagram, it can be seen that after the user sends an operation request by using the model module in the MVC architecture, the system can call the user's specific operation request by using the view module, and at the same time feed back user event information to the controller. The controller will further retrieve the processing task data in the model module, and display the feedback and specific content information retrieved to the system user through the view module [1–6] It can greatly satisfy the effective management of the current university teaching system.

### 2.2. Genetic Algorithm

#### 2.2.1. Basic Mathematical Model

The basic genetic algorithm consists of 8-tuples in the following formula, namely:

(1) $$\begin{array}{c} SGA=\left(C,E,P_{0},M,\Phi ,\tau ,\psi ,T\right). \end{array}$$

In formula (1):

*С*-represents the individual coding method (binary), which is the basic factor in genetic algorithm. A combination formed by the connection of genes and chromosomes is a solution for curriculum arrangement;

*Е*—— represents the fitness evaluation function of the individual. Use this function value to distinguish whether the individual meets the requirements; P0-represents the initial group, a combination of courses randomly formed by genetic algorithm, and subsequent optimization of genetic algorithm will be carried out around the initial group;

*М*——represents the size of the group;

Ф——represents the selection operator, and the calculation method is filtered by the fitness value. Generally, the larger the value, the easier it is to be selected;

г——represents the crossover operator. The new individual is generated by the random exchange of genes from the parent individual, and the single point crossover method is adopted;

*ψ*-represents the mutation operator, the parent individual randomly changes the individual's own gene value, and adopts a single point mutation of the gene;

*Т*——represents the termination condition of the algorithm. When performing genetic iteration, we generally set a certain parameter value, and the operation is terminated when the parameter is iterated algebraically [7].

#### 2.2.2. Operation Process

When using genetic algorithms to develop a hybrid teaching system, follow the steps below:

1. Choose an appropriate way to encode system parameters, and convert the relatively optimized solution set into chromosomes for representation;
2. Determine the initial group of the system;
3. Define the fitness function;
4. Genetic operation of the design system;
5. Control the setting of parameters such as the size of the population and the probability of genetic manipulation;
6. Judge whether the generated group meets a specified index, if it is satisfied, exit the calculation, if it is not satisfied, return to the operation of calculating the fitness function value [8]. The specific flow chart is shown in Figure 2.

## 3. System Design of Mixed Teaching Mode

### 3.1. System Architecture Design

In order to facilitate the system to have stronger scalability and maintainability, in the process of architecture selection, the MVC architecture is finally selected as the system architecture of the college online teaching management system, combined with specific design, the entire college online hybrid teaching management system The detailed design of the overall architecture is shown in Figure 3.

The overall architecture of this hybrid teaching management system is mainly composed of the presentation layer, the system service layer and the data layer. The presentation layer is mainly used to provide access interfaces for system users of the university hybrid teaching management system. Through the front-end operation interface of this layer, users can provide interface services for various business operations in the system service layer [9].

The system service layer is mainly composed of core business and business support parts. The core business part specifically includes the operation of system management, online learning management and other business functions. At the same time, in order to provide strong support for the main core business operations, in this layer The business support part has designed user authority configuration and information query and information exchange services.

The data layer is mainly used to provide services for the retrieval and storage of all data information in the hybrid teaching management system of colleges and universities, and to provide data support for the smooth progress of various core businesses in the system service layer. The business functions to be realized mainly include a variety of data information such as online course information database and video-on-demand course information database [10, 11].

### 3.2. System Network Topology Design

By combining the overall architecture of the system, it can be seen that the entire university hybrid teaching management system mainly adopts the MVC three-tier architecture. In order to meet the characteristics of the scattered users of the system combined with the characteristics of the system architecture, the specific network topology structure diagram of the university hybrid teaching management system The design is shown in Figure 4.

It can be clearly found that in the course of business operation of the college hybrid teaching management system, all users in the system can use the external network and the college intranet for system login access, and the terminal devices used are computers. The network architecture can be divided into the core area and the gatekeeper isolation area. For the core area, its firewall can effectively guarantee the security performance of the system. The main method is the connection between the load balancing server and the gatekeeper isolation area, thereby providing access to the database in this area. Manage and control servers and application servers [12–14].

### 3.3. System Function Module Design

Online learning management is an important module of the entire university's hybrid teaching management system. It is mainly used by teachers to create, review and publish online courses. College students can also use this function for online course inquiry and registration. Combined with actual needs, the design of the functional structure diagram of the specific online learning management module is shown in Figure 5. The entire online learning management module mainly includes three sub-functions: online course management, my course management, and online learning.

The online course management sub-module is composed of two main functions: online course creation and online course review and release. The entire course management sub-module is composed of three main functions: online course inquiry, online course registration, and my course inquiry. By combining the actual needs and target requirements of the college, students can use this module to query relevant course information and combine The training goal requires course application and registration, and at the same time, it is possible to inquire in detail about the course status declared by the individual. The online learning sub-module is composed of three main functions: course study material management, course video on demand, and online interaction. In combination with the online learning function requirements, the detailed online learning data management work sequence diagram is shown in Figure 6. For the various video materials uploaded by users, the system administrator is responsible for categorizing them and sorting them according to the number of views. At the same time, they set tags for each video so that users can easily and quickly find what they need through search and other means. Video learning, in the search process, on the one hand, the system administrator can combine with the actual situation to directly query the ranking of the popular course videos, on the other hand, it can also directly search through the input of the course keywords. When students are learning on video-on-demand, they can use the interactive module to leave a message and ask questions at any time, and the teacher in charge can answer questions through the interactive platform after seeing the student's message [15].

Combined with the working sequence diagram of the hybrid teaching management system, it can be known that the system operator clicks “online learning management” on the operation homepage, then enters “online learning,” and then completes the specific creation of the course video materials according to actual needs, and completes the course video Upload and edit on-demand resource information. After the operation is completed, after the course video on-demand resource information database is updated, college students can search for course video-on-demand resources. After entering the required query on-demand resource keywords, the system will combine the input keywords The matching information is screened in the database, and then the qualified resource information is displayed. In the process of watching the on-demand video, the college students can enter the interactive information of the course.

### 3.4. System Database Design

The database logical structure design is the design of the overall logical structure of the database. The design methods mainly include top-down, bottom-up and one-by-one Three kinds of expansion. Among them, the top-down is mainly through the design of the overall data structure, and then gradually refines until the design of the entire data structure is completed; bottom-up merges the data structure according to the logical relationship between the data, until the overall data structure is completed the design of. Combining the detailed design of the overall E_R diagram of the university hybrid teaching management system and the specific data logic structure rules, the design of the main data information tables such as online course information, test paper information and basic learning file information included in the system is explained.

For a detailed description of the online course information table, see Table 1. According to the design of the online course information table, combined with the corresponding data logical structure, this information table is composed of course name, instructor, course hours, course credits, and course duration.

## 4. Implementation of a Hybrid Teaching System Based on Deep Learning

### 4.1. System Implementation Environment

After completing the design of the functional modules and database of the hybrid teaching management system in universities, it is necessary to combine the detailed design of the system to design and implement the operation interface of each functional module of the system, combine the detailed design of the system, and control the system through the front-end operation interface. The specific implementation is fully demonstrated. In the implementation process, the corresponding hardware and software are required to support. In order to meet the stable and reliable operation of the implementation interface, the hardware and software configuration of the development side and the server side required for the system implementation are required:

1. Development end hardware and software configuration
2. On the development side, in order to facilitate the debugging of the entire college online teaching management system, in the process of selecting the terminal on the development side, the main terminal processor selected is i7-9750H, six-core CPU, memory capacity of 32GB, and hard disk type SSD. The size of the solid state drive is 1TB, and the main choice for software development is Eclipse 5.0.
3. Server hardware and software configuration
4. On the server side, combined with the requirements of system development, the server side supports RDIMM/LRDIMM, with a minimum memory of 64GB, with data protection functions such as encrypted signature firmware, secure boot, system lock, and secure erasure. Oracle is selected in the selection of database software 11g version database.

### 4.2. Implementation of the Mixed Teaching Management Module

Combined with the actual function design, the entire blended learning management module mainly includes three sub-functions: online course management, my course management, and online learning materials. The detailed design of the class diagram of the online learning management module is shown in Figure 7. Combined with the class diagram of the online learning management module, the entire Online Learning Management Class is mainly associated with three sub-categories: Online Course Management Class, My Cours Management Class, and Online Learning Materials Class. Among them, the Online Course Management sub-category mainly includes online Course Creation () And online Course Audit and Publication () two operation methods, used to realize the creation, review and publication of Online Course Information; My Course Management Class subclasses include online Course Query (), online Course Registration () and my Course Query () Three methods, using the My Course Management interface to implement online course query and registration and other related operations, and can be correlated with Online Course Information in the Online Course Management class; Online Learning Materials Class subclasses include course Data Management (), Course Video on Demand Learning() and online Learning Interaction() three operation methods are used to realize the management of VOD Resource Information, and use the Online Learning Interaction interface to realize the function operation of video-on-demand course information query and online interactive learning.

Combined with the specific design, the implementation of the operation interface of the online course management sub-functions in the blended learning management module is shown in Figure 8. From the online course management operation interface, it can be seen that the instructor can create the online courses he is responsible for, such as the specific courseware of the course, after-school exercises, and real test models.

The realization of the core code of the personal information management operation part in the management module of the entire hybrid teaching management system is shown in Figure 9 below:

### 4.3. System Test

#### 4.3.1. Function Test

In the process of testing the online learning management module, detailed and comprehensive tests were mainly conducted on the related operations of online course management, my course management, and online learning. The specific online learning management module test case descriptions are shown in Table 2. From the online learning management function test case, it can be seen that in the process of testing the online learning management function, the main functions of online course management, my course management and online learning are comprehensively tested, and the actual test results can meet the expected indicators and Require.

#### 4.3.2. Performance Test

In the process of testing the performance of the entire university hybrid teaching management system, the author mainly conducts the performance of concurrent users of the entire system. The detailed test situation is shown in Figure 10. It can be seen from the concurrent performance test of the user login and processing flow that, combined with the actual performance requirements of online teaching in colleges and universities, in the specific test, the number of concurrent users selected is 300, and the main tool used in the test process is LoadRunner for testing. According to the concurrent performance test, the detailed test situation analysis table is shown in Table 3. It can be seen from the test situation analysis table that when the maximum test user is 300 people, the actual test response time is 4.941 seconds, and the expected performance index can be met within the expected response time.

## 5. Conclusion

Based on the current situation of mixed teaching management, this paper attempts to design and develop a set of mixed teaching management system suitable for colleges and universities, realizes the informationization of college daily management, and solves the problems of low efficiency and high error rate of traditional manual management mode. By using the MVC architecture and Oracle database and other major technologies, the author has mainly completed the following aspects: [16–24].

1. A detailed analysis of the business requirements for the application of the hybrid teaching management system in colleges and universities is carried out, and the business functions required by the hybrid teaching management system in colleges and universities as well as the specific functional requirements and performance requirements of the system are proposed.
2. According to the specific design and implementation, the system function test and system performance test are completed by equivalence class division and boundary value analysis methods, and the test results can meet the expected index requirements.

The college hybrid teaching management system designed in this article still needs to be improved. For example, although the online learning management module already has the interactive function of online learning, it only realizes simple text communication. It is not possible to directly communicate with the instructor for the time being. Group discussions, etc., still need to be further improved.

## Figures and Tables

**Figure 1:** MVC architecture diagram.

**Figure 2:** Flow chart of genetic algorithm.

**Figure 3:** System overall architecture diagram.

**Figure 4:** Network topology structure diagram of the hybrid teaching management system in colleges and universities.

**Figure 5:** Functional structure diagram of online learning management module.

**Figure 6:** Working sequence diagram of online learning operation.

**Figure 7:** Class diagram of online learning management module.

**Figure 8:** User login implementation interface.

**Figure 9:** The core code of the management module of the hybrid teaching management system.

**Figure 10:** System concurrent performance test.

**Table 1:** Detailed description of online course information table.

Field name	Field type and length	Field explanation
Course_ID	Varchar2(20)	Course number (primary key)
Course_Name	Varchar2(50)	Course title
Course_Type	Varchar2(30)	Course type
Teacher	Varchar2(20)	Teacher
Course_Hours	Float(10)	Course hours
Chapter_Content	Varchar2(2000)	Chapter content
Course_Credit	Float(10)	Course credits
Subordinate_Specialty	Varchar2(50)	Their profession
Course_Manager	Varchar2(20)	Course manager
Exercise	Varchar2(2000)	Homework
Course_Duration	Float(10)	Course duration

**Table 2:** Online learning management function test case description table.

Functional test number	Testing requirements	Prerequisites	Detailed operation	Expected outcome	Results of testing
GN-003	Able to realize online course creation and online course review and release operations in the online course management sub-module	Use the identity of the instructor in school Click “Online Learning Management” in the main interface of the online teaching management system to enter smoothly	On the main interface of the displayed system, select “Online Learning Management Selection” and “Online Course Management”	Successfully enter the “Online Learning Management” page, select “Online Course Management,” select the corresponding course template, and click Create. After the specific content of the online course is successfully created and imported, the database information can be updated, and prompts will be given. Wait approved, the specific content of the course can be	Pass through

GN-004	Able to realize online course query and registration in the sub-module of my course management	Use the status of a college student to click “online learning management” in the main interface of the school's online teaching management system to enter it smoothly	On the main interface of the displayed system, select “Online Learning Management Selection” and “Then My Course Management”	successfully released, and can be inquired on the system homepage Successfully enter the “Online Learning Management” interface, select “My Course Management,” you can query the published online courses according to the release date or course name, and can declare the course as a student. After the registration is successful, the system can prompt to sign up success	Pass through

GN-0 05	Able to realize the video-on-demand and learning operation of the course in the online learning sub-module	Use the status of a college student to click on “Online Learning Management” in the main interface of the online teaching management system to enter it smoothly	On the main interface of the displayed system, select “Online Learning Management Selection” and “Then Online Learning”	Successfully enter the “online learning management” interface, select “online learning,” you can query the selected course video in the displayed interface, and can order the required learning video according to the date and chapter, and the system can play the selected video normally, during the learning process, be able to mark the videos you watched and make corresponding notes	Pass through

**Table 3:** Concurrent user performance test table.

Number of test users	Expected test value (seconds)	Actual test value (seconds)
50	2.0	1.444
100	3.0	2.688
150	4.0	3.676
200	5.0	4.941

## Data Availability

The dataset can be accessed upon request.
